The article "Data Analysis for Modeling the Effect of Acupuncture on Postchemotherapy Cancer Fatigue in Gynecologic Oncology Patients" was retracted in 2023. Reasons: signs of a paper mill; suspected computer-generated content; unreliable results or conclusions; lack of ethics approval or compliance.

# Data Analysis for Modeling the Effect of Acupuncture on Postchemotherapy Cancer Fatigue in Gynecologic Oncology Patients

**DOI:** 10.1155/2022/7201485

**Published:** 2022-06-13

**Authors:** Jili Deng, Yao Qian, Xingyu Chen, Juan Jiang

**Affiliations:** ^1^Clinical Medical College, Guang'an Vocational & Technical College, Guang'an, Sichuan 638500, China; ^2^Cancer Hospital of Chongqing University, Shapingba, Chongqing 400030, China

## Abstract

Now cancer-related fatigue is gradually being emphasized, which is a common symptom in cancer patients. During long-term radiotherapy, the emotion of patients will be affected directly, and inevitably produce cancer-caused fatigue needle symptoms. Moreover, the weakness and fatigue are always produced simultaneously, which are harmful to patients' prognosis level of their overall survival quality. The acupuncture has a helpful effect on improving the Chinese medical evidence of side effects caused by radiotherapy and chemotherapy in tumor patients. In this paper, we model the effect of acupuncture on cancer fatigue after chemotherapy in gynecologic oncology patients through data analysis, so as to effectively analyze the degree of cancer fatigue after chemotherapy in patients.

## 1. Introduction

Cancer-related fatigue (CRF) is a series of subjective feelings resulting from prolonged pain and stress caused by cancer and its related treatments, an emotional or cognitive fatigue that often manifests as a persistent feeling of exhaustion that is disproportionate to recent activities and interferes with the patient's normal functioning, with a reported incidence of CRF in patients receiving treatment of CRF has been reported to occur in 52–90% of treated patients [1], with 9–45% of patients experiencing moderate-to-severe CRF, and CRF can persist months or even decades after the end of cancer treatment [2, 3]. Current research on the pathogenesis of CRF has focused on inflammation, central nervous system (CNS) disorders, and mitochondrial dysfunction, and CRF is highly harmful and difficult to cure in the long term, with a dual negative impact on patients' physical and psychological health. Current therapies have not shown sufficient advantages in changing cancer-related symptoms (e.g., anemia, cachexia, depression, and sleep disorders), while research on acupuncture to improve tumor-related symptoms (e.g., pain, vomiting, persistent eructation, and dry mouth) is flourishing, and its role in relieving cancer fatigue is continuously proven and gradually applied in clinical practice [4]. The main mechanism of its good protective effect on the chemotherapy body is that acupuncture can improve the body's immune function and antagonize the side effects of chemotherapy drugs [5].

In the *Nei Jing*, there is a view that if the righteousness of the qi exists inside the body, the evil cannot dry it out, and the qi of the evil will be deficient, and the system that can resist the invasion of internal and external disease and evil is classified as the righteousness. The immune system of the body belongs to the positive qi, so it is especially important for tumor patients, especially for patients undergoing chemotherapy, to improve the immune system by supplementing the positive qi. In this study, from the perspective of TCM, the key to treatment is to regulate the qi of the five organs, and also to nourish the qi and blood [6]. The selected acupuncture points play a role in tonifying the kidneys and benefiting qi and regulating yin and yang. The second is to perform acupuncture techniques, from the streak of Nei Jing, through the summary and refinement of generations of doctors, has formed a relatively complete system, such as xu shen mending diarrhea, open and close mending diarrhea, twisting mending diarrhea, breathing mending diarrhea, as well as burning mountain fire through the days of cold and other techniques [7]. In clinical practice, the author found that traditional acupuncture techniques have obvious advantages over electroacupuncture and often receive good results with nutrition and psychological guidance. Chinese acupuncture is good at regulating the overall function and has unique advantages in clinical treatment, so it has good application prospects in the field of CRF treatment [8].

American ginseng is a drug that has been identified to alleviate cancer-caused fatigue. Although acupuncture is not the traditional treatment of choice for the relief of oncogenic fatigue or postchemotherapy fatigue, its effectiveness and affordability still make its widespread clinical use possible [9]. Based on abovementioned points, this study use data analysis method to model the effect of acupuncture on postchemotherapy cancer fatigue in gynecologic oncology patients, so as to target and improve patients' postoperative recovery.

## 2. Related Work

Gynecologic tumors are one of the most common causes of death in gynecologic patients, and epidemiology shows that the mortality rate of this disease is up to about 50% in the middle and late stages, and its incidence is increasing year by year and tends to be younger [10]. The current treatment modalities are based on the benignity and malignancy of gynecologic tumors and the stage of the disease. Early stage patients are treated with resection and debulking, and terminal-stage patients are treated with hysterectomy combined with radiation therapy to reduce the risk of recurrence or distant metastasis [11]. However, with the prolonged duration of radiotherapy, most patients are prone to mental weakness, fatigue, and negative treatment under the influence of life and physiology, which interferes with the clinical efficacy.

Although the mechanism of the effect of acupuncture in the treatment of this disease is not clear, some studies have shown that acupuncture and its related therapies (such as auricular acupuncture and warm acupuncture) have great potential as an adjuvant therapy to alleviate CRF in patients and improve the quality of survival of patients, and the clinical studies of acupuncture and its related therapies in recent years are summarized, analyzed, and summarized as follows. A randomized double-blind controlled trial was conducted by [12], which included 28 patients with CRF of lung cancer, with acupoints selected as 45 min/time, 2 times/week, and continued treatment for 4 weeks with a 2-week follow-up, while the sham acupuncture group took the same acupoints but without needles into the skin [13].

In [14], authors divided 302 patients with breast cancer CRF into treatment group and waiting group in the 3 : 1ratio. In addition to conventional care, the treatment group was combined with acupuncture intervention, with acupuncture points selected as Feet Three Miles, Sanyinjiao, and Hegu, and if patients had upper-limb edema, the Hegu point could be changed to Yanglingquan, and Yinlingquan for 20 min/time, once/week for 6 weeks. Researchers in [15] used moxibustion to treat CRF patients, and the treatment group used moxa suspension method, with acupoints selected from the foot three li, blood sea, taixi, hanging bell, qi sea, and guan yuan, each acupuncture point moxibustion for 10–20 min, 1 time/d, 4 weeks as a course of treatment.

Using spaced ginger moxibustion as a treatment in [1], 40 patients with CRF were included in a single-arm trial, and spaced ginger moxibustion was administered at the foot San Li point in these patients for 20–30 min/concussion, 3 cones/time, 1 time/d for 10 d. The results showed that after spaced ginger moxibustion at the foot San Li, the PRFS scores of patients with CRF were lower in all dimensions than before treatment (*P* < 0.05). They studied 120 patients with CRF of intermediate-to-advanced lung cancer in [16], and both groups used conventional interventions, and then the treatment group was combined with thermal moxibustion intervention. The total RPFS score and each dimension score of the study group were significantly lower than the control group (*P* < 0.05), and the total efficacy rate of Chinese medical evidence was 81.7% in the treatment group and 46.7% in the control group, indicating that thermal moxibustion, in addition to improving the degree of fatigue can also improve the immunity of the body and improve the systemic symptoms of patients.

A total of 46 patients were included in [17] with CRF after chemotherapy, randomly divided into control and treatment groups, the control group was given symptomatic treatment, and the treatment group was treated with mai gong moxibustion for 10 d starting from 3 d before the current cycle of chemotherapy, with mai gong moxibustion on both sides of the third mile of the foot, 1 time/d, 7 strokes per point. The results showed that the mai gong moxibustion group was better than the control group in relieving the degree of CRF, increasing hemoglobin, and improving patients' clinically. The results showed that the moxibustion group was better than the control group in relieving CRF, increasing hemoglobin and improving clinical symptoms (*P* < 0.05), and significantly reducing the toxic side effects of chemotherapy.

A randomized controlled trial was conducted on 78 cancer patients with CRF [18]. The control group was given conventional care and aerobic exercise, the observation group was given auricular acupoint pressure dou, selected liver, spleen, stomach, Shenmen, and jiao-sense for pressure. Each point was pressed 4–6 times, 3–5 min/time, and each time the pressure was applied to one side of the auricular point, after 3 d, it was changed to the other side of the auricular point, alternating between the two ears.

## 3. Strategies for Data Analysis of the Effects of Cancer Fatigue

The core of data analysis based on the effect of acupuncture on cancer fatigue after chemotherapy in gynecologic oncology patients lies in how to determine the amount of influence needed to be given for the current error from the input data and control data collected historically. The process of solving this problem can be decomposed into two steps: the first step is to map the historical collected control quantities to the error values one by one, and the second step uses a trained control algorithm to predict the amount of control required to give the current error value. The characteristic of this approach is that there is no need to determine the actual mathematical model and model properties of the system, and the function of modeling the effect of acupuncture [19] on cancer fatigue after chemotherapy in gynecological oncology patients can be achieved using only the inputs and outputs of the system.

The above scheme is the algorithmic idea of an artificial neural network. A neural network relies on many neuron models, which pass each other through connections with weights. When all the inputs received by a neuron break through the activation function, the neuron will release the output, which is the classical “M-P neuron model.” Numerous individual neurons are connected in a particular way to form a multilayer neural network. When the activation characteristics are satisfied, the lower-level neurons will output to the higher-level neurons to induce higher-order statistical characteristics layer by layer.

Traditional data analysis techniques require modeling the observation environment, building a model by observing the system, then testing the stability and validity of the model with measured data, and finally analyzing all new data with a fixed model. This model is often difficult to maintain in a stable state due to the errors and disturbances in the actual use. The strategy of artificial neural network is completely opposite, after learning a large number of input and output signals, the network will analyze a new data and give appropriate output values, and errors and disturbances can be added to the learning of the network, making the network effectively discriminate between actual input signals and policy errors and disturbances.

After learning the historical data and disturbances, the system is tested using new data to continuously correct the output of the artificial neural network. In modeling the effect of acupuncture on postchemotherapy cancer fatigue in gynecologic oncology patients, a set of errors and controls of actual versus set quality for sampling statistics performed over a fixed period of time constitutes a set of input-output pairs, while a database consisting of a large number of input-output pairs constitutes the training samples for the neural network. Training against these samples requires stable learning rules.

One of the most representative neural network algorithms is the error back propagation algorithm (BP). As mentioned above, each neuron in a neural network needs to be connected to each other by some rules, and this connection is called the hidden layer in the neural network. In the case of Is output, the signal is passed to each neuron in the output layer as input, which forms a forward propagation process intact, and when the actual output is in error compared with the theoretical value, it enters the reverse propagation stage. By calculating the error between the output value and the theoretical value, the error and weighting value of the neurons in each layer are gradually corrected from the output layer in the direction of the input layer until they match the data in the input layer, which forms a cycle of the BP algorithm. By continuously correcting this neuron error and connection weighting, the learning effect is achieved until the error value is reduced to a preset target. The time rate of this algorithm is constant; more data means more learning cycles, and more data and learning cycles also mean more correction processes, that is, the longer the learning time, the slower the convergence rate. Therefore, in the face of large-scale data, the BP algorithm has the characteristics of time-consuming and slow response, and this method is obviously not applicable in the flow control process that requires real-time response. On the other hand, the determination of the weighting value is a gradual convergence process, and even when converging to a certain determined value, it does not mean that this value is globally minimized relative to the error plane, thus falling into a local optimum.

To address these two problems, the improvement direction of the algorithm strategy can be determined as reducing the training time and increasing the test accuracy. The Extreme Learning Machine (hereinafter referred to as “ELM”) is another new feedforward neural network model proposed in recent years, which adopts the method of random input weighting and hidden-layer partials, treating the system as a linear model by solving the generalized matrix method. Seeing the system as a linear model, the output weights are obtained by solving the generalized matrix, which eventually converts the problem into a simple linear regression algorithm, thus greatly reducing the training time, and its basic representation is

(1) $$\begin{array}{c} t_{j}=\sum_{i=1}^{N}\beta_{i}g_{i}\left(x_{j}\right)\\ =\sum_{i=1}^{N}\beta_{i}g_{i}\left(w_{i}x_{j}+b_{i}\right),\;\left(j=1,2,\ldots ,N\right), \end{array}$$

where *t*_*j*_ is the output of model; *N* is the number of hidden layer; *β*_*i*_ is the weight matrix of output; *g*_*i*_ (·) is the activation function; *w*_*i*_ is the input weight; *x*_*j*_ is the input; *b*_*i*_ is the bias of hidden layer.In matrix form it can be expressed as follows:

(2) $$\begin{array}{c} HB=T. \end{array}$$

In equation (2), *H* is the state matrix that will contain a neuronal network with 100 hidden layers.

Expanded as follows:

(3) $$\begin{array}{c} H=\left[\begin{array}{ccc} g\left(w_{1}x_{11.1}+b_{1}\right) & \cdots & g\left(w_{100}x_{11.9}+b_{100}\right)\\ \vdots & \ddots & \vdots \\ g\left(w_{1}x_{n.m}1+b_{1}\right) & \cdots & g\left(w_{100}x_{nm.9}+b_{100}\right) \end{array}\right]. \end{array}$$

The expression of the output-weighting matrix *β* is defined as follows:

(4) $$\begin{array}{c} \beta ={\left[\beta_{1},\ldots ,\beta_{100}\right]}^{T}. \end{array}$$

When the training data set is fed into the neural network of ELM hidden layer, the state transfer matrix *H* is obtained and the inverse matrix *β* is derived, and the learning stops when the training reaches a preset number of times or the error is reduced to a preset range.

Unlike the BP algorithm, ELM randomly selects the weighting values between the input and hidden layers and the deviation values of each neuron in the hidden layer, which significantly improves the learning efficiency and reduces the training time. The number of neurons (#neurons) in the hidden layer needs to be increased accordingly to guarantee in the accuracy of the output due to the random selection of parameters between the input layer and the hidden layer. In this way, the nonlinear system is simplified to a linear system solution.

The results obtained using ELM are shown in Table 1, after learning 400 sets of input and output data and testing with reference to 20 sets of data.

As shown in Table 1, ELM only needs little training time to guarantee high-learning accuracy, but the test accuracy is low, and the algorithm needs to be improved.

ELM's characteristic of randomly selecting weighting values between input layers to hidden layers, many nonessential inputs instead enter the hidden layers with higher weighting values, making it more difficult to correct the deviation values in the next layers, and the number of layers of hidden layers and #neurons in hidden layers need to be continuously increased to improve the accuracy. Therefore, making the algorithm find the optimal path and optimal parameters in the hidden layer accurately and get the optimal solution is an important entry point to improve the test accuracy, that is, solving the combinatorial optimization problem [4].

Simulated annealing algorithm is a global search algorithm that can effectively avoid the algorithm from stagnating in the local minimum or maximum and is a classical algorithm for solving combinatorial optimization problems. A large value *t* is first given, and the solution *i* is randomly derived as the initial solution. Given *t* and then a randomly derived solution *j*, *j* ∈ (*N*_*i*_), and *Ni* is the domain of *i*, the transfer probability from solution *i* to *j* is

(5) $$\begin{array}{c} P_{t}=\left(i\Rightarrow j\right)=\left\{\begin{array}{cc} 1, & f\left(j\right)<f\left(i\right),\\ e^{f\left(j\right)-f\left(i\right)/t}, & \text{other.} \end{array}\right. \end{array}$$

If solution *j* is accepted, it becomes the new solution instead of solution *i*. Otherwise, the original solution *i* is retained, and the process is repeated until it equilibrates under the control parameter *t*. After a sufficient number of state transfers, the control parameter *t* needs to be slowly decreased, and then the above process is repeated under the new parameter *t* until the parameter *t* is decreased to a small enough size, and the final result is an optimal solution to the combinatorial optimization problem. The pseudo code of the algorithm is as follows:

The simulated annealing algorithm is a typical two-level, nested-loop structure to achieve global search by random solving. In such an algorithm, some solutions which are close to the indicator function are randomly accepted. Therefore, it is impossible to find the optimal solution in a short time. But with the decrease of control parameter *t,* the probability of finding the optimal solution rises.

ELM determines each parameter of the algorithm by training the training data, and the difference in the parameters determines the magnitude of the accuracy. Therefore, the selection of parameters can be optimized by using the global search property of the simulated annealing algorithm. The improvement steps of ELM using the simulated annealing algorithm are described here.

First, the indicator function *f*(*i*) is given. Here the variance of the training samples is evaluated as the indicator function to represent the error level more appropriately, that is,

(6) $$\begin{array}{c} f\left(i\right)=E=\frac{1}{2p}\sum p\sum k{\left(t_{k}^{p}-o_{k}^{p}\right)}^{2}. \end{array}$$

The preset error is less than or equal to *E*_*m*_, and the decline factor *a*  = 0.97, then the parameter *t*_*k*+1_=*at*_*k*_.

Initialize the network weighting and bias values, that is, *W*=(*ω*, *β*)=(*ω*_1_,…, *ω*_*d*_; *β*_1_,…, *β*_*d*_), where *ω* is the weighting value on the neuron connections, and *β* is the output weighting value. Make the initial solution *i*=*W*, and the resulting solution is *i*=(*ω*_1_^*∗*^,…, *ω*_*d*_^*∗*^; *β*_1_^*∗*^,…, *β*_*d*_^*∗*^). The optimization can be completed by using it as the new weighting value and adding it to ELM. By this method, the BP algorithm and ELM method are improved, respectively. A total of 400 sets of input and output data are learned and tested with reference to 20 sets of data, and the results are shown in Table 2.

The data results in Table 2 intuitively show that after the simulated annealing algorithm was chosen to improve the parameters of the two learning methods of the neural network, and the test accuracy was significantly improved. The test accuracy of the BP algorithm was better than ELM method, but the training time was significantly longer and might not match the actual usage scenario.

## 4. Case Study

For investigating the role of acupuncture as an adjunctive treatment measure in alleviating cancer fatigue after chemotherapy for gynecologic tumors patients who were hospitalized in the gynecologic oncology department for more than three courses of chemotherapy from June 2012 to September 2013 were selected. A total of 120 patients, aged 16 to 70 years with a mean of (52 ± 3.3) years, who had fatigue assessed at level 2 or higher by the Brief Fatigue Inventory (BFI), were pathologically confirmed to have ovarian cancer in 50 cases, cervical cancer in 42 cases, and endometrial cancer in 28 cases, and all received chemotherapy with TP (paclitaxel combined with nedaplatin) regimen. A simple randomization method was used to generate random numbers using PEMS3.1 statistical software. When eligible cases were entered into the trial, patients were assigned to 40 cases in each group, including the experimental, drug, and blank group in the randomized number table in the order of specific inclusion. The results are shown in Table 3.

Exclusion criteria: those with other serious physical diseases; those with psychiatric diseases; those with serious intellectual or cognitive impairment; those with serious chemotherapy side effects and impairment of heart, liver, kidney, and other important organ functions; those who discontinued or stopped treatment during the treatment period [20–22].

In the experimental group, acupuncture was used: acupoints were taken from Zhongguancest, Neiguan, Fusanli, Sanyinjiao, Qihai, Guangyuan, Kidney Yu, and Liver Yu. The acupuncture technique was a combination of lifting and twisting, and the method of flat tonification and flat diarrhea was used. After acupuncture, warm needle moxibustion was applied to foot San Li, Qi Hai, and Guan Yuan with 2 cm long moxa cones for two strokes.

Self-assessment of fatigue was performed by the BFI. BFI to self-assess their fatigue status and observe the changes in the scores of the three groups after two courses of treatment. The total symptom scores of the two groups were compared, and the improvement rate of symptom scores was calculated. The improvement rate of points ≥70% was considered effective, the improvement rate of points ≥30% was considered effective, and the improvement rate of points <30% was considered ineffective [23–25].

The difference between the fatigue levels of the three groups before chemotherapy was not statistically significant (*P* > 0.05), but after chemotherapy (day 3), their fatigue levels were significantly higher (*P* > 0.01). Although there was no significant advantage in the acupuncture intervention group compared with the western ginseng group (*P* > 0.05), it also showed the effectiveness of acupuncture intervention (shown in Table 4).

The points of patients in both experimental and drug groups decreased compared with those after chemotherapy (*P* < 0.01), and there was a tendency for acupuncture treatment to improve the points. The results are displayed in Table 5.

The improvement of TCM symptoms in both the experimental group and the drug group is much better than that in the blank group (*P* < 0.01), which is shown in Table 6.

All patients were pathologically confirmed as gynecologic tumors, and the control group was treated with conventional chemotherapy, that is, TP therapy (paclitaxel combined with nedaplatin); the observation group was adjuvantly treated with acupuncture and moxibustion, taking the patient's acupuncture points of Zhongsanli, Foot Sanli, Neiguan, Sanyinjiao, Qihai, Guanyuan, Kidney, and Liver. After such operations, warm acupuncture was applied with 2 cm long moxa cones with 20 min, once a day, three times a week of treatment.

The data recorded in the study were processed and analyzed using the statistical software SPSS17.0., and the results as shown in Table 7.

The experimental group started acupuncture treatment on the first day of chemotherapy, once a day, three times a week for 3 weeks. The drug group started oral western ginseng, 2000 mg/day, three times daily for 3 weeks. No other interventions were given to the blank group. The patients in the three groups were evaluated by BFI and TCM syndrome evaluation before chemotherapy, on the third day of chemotherapy (after chemotherapy), and 3 weeks of chemotherapy (after treatment), respectively, and the evaluation results were compared.

The overall fatigue levels of the patients in the three groups were comparable before chemotherapy, and there were no significant differences in the BFI assessment and TCM syndrome scores (*P* > 0.05); after chemotherapy, the patients in all three groups increased significantly (*P* < 0.01); after treatment, the above scores of the patients in the experimental group decreased significantly (*P* < 0.01).

## 5. Conclusion

In this paper, we model the effect of acupuncture about cancer fatigue after chemotherapy in gynecologic oncology patients based on data analysis method. By comparing the different results of patients' cancer fatigue BFI scale scores in two periods, acupuncture treatment can significantly improve cancer fatigue. Although there is no significant advantage compared with oral western ginseng method, its effectiveness may make acupuncture to be a reliable adjuvant treatment for cancer fatigue. In the future, the clinical trial data, the trial design, and the corresponding reports of multicenter, randomized, controlled clinical trials are consider to make a reliable clinical decision of acupuncture treatment.

## Figures and Tables

**Algorithm 1:** Global search

**Table 1:** ELM algorithm learning test results.

ELM algorithm			
Learning phase		Test phase	
Learning accuracy (%)	97.66	Test accuracy (%)	86.68
Training time (s)	0.04		

**Table 2:** Improved BP algorithm and ELM learning test results.

SA-BP algorithm		SA-ELM algorithm	
Learning accuracy (%)	98.55	Learning accuracy (%)	99.32
Training time (s)	40.99	Training time (s)	0.79
Test accuracy (%)	95.01	Test accuracy (%)	94.01

**Table 3:** Comparison of basic materials among the three groups.

Group	*n*	Age	PS score			Tumor type				Pathological stage				Number of chemotherapy	
			0	1	2	Cervical	Ovarian	Endometrial	Other	I	II	III	IV	3	4∼6
Experience	40	51 ± 5.3	11	19	10	16	21	7	0	12	12	15	1	19	21
Drug	40	52 ± 3.6	9	22	9	13	15	14	1	7	13	15	5	17	23
Blank	40	53 ± 6.5	8	25	7	10	17	9	0	14	9	17	0	18	22

**Table 4:** Comparison of comprehensive fatigue level.

Group	*n*	Before chemotherapy	After chemotherapy	After treatment
Experience group	40	4.31 ± 0.6	7.01 ± 0.5^*∗∗*^	3.55 ± 0.6^*∗∗*##ΔΔ^
Drug group	40	4.61 ± 0.2	7.81 ± 0.2^*∗∗*^	3.51 ± 0.8^*∗∗*##ΔΔ^
Blank group	40	4.89 ± 0.7	6.19 ± 0.3^*∗∗*^	6.01 ± 0.3^*∗∗*##ΔΔ^

Note. Compared with before chemotherapy, ^*∗∗*^*P* < 0.01; compared with after chemotherapy, ^##^*P* < 0.01; compared with the same period in the blank group, ^ΔΔ^*P*.

**Table 5:** Comparison of Chinese medicine evidence scores.

Group	*n*	Before chemotherapy	After chemotherapy	After treatment
Experience group	40	10.31 ± 0.6	17.09 ± 0.5^*∗∗*^	7.72 ± 0.3^*∗∗*##ΔΔ^
Drug group	40	14.31 ± 0.3	19.81 ± 1.2^*∗∗*^	8.51 ± 0.2^*∗∗*##ΔΔ^
Blank group	40	12.89 ± 0.2	19.19 ± 0.3^*∗∗*^	17.32 ± 0.3^*∗∗*##ΔΔ^

**Table 6:** Comparison of improvement of TCM symptoms.

Group	*n*	Remarkable effect	Effective	Invalid	Total effective rate (%)
Experience group	40	26	11	3	91.9
Drug group	40	28	9	6	88.7
Blank group	40	0	8	32	16.8

**Table 7:** Comparison of Chinese medicine symptoms scores and cancer fatigue BFI scores $\left(\bar{x}\pm s\right)$.

Group	BFI		TCM syndrome	
	Before treatment	After treatment	Before treatment	After treatment
Control group (*n* = 35)	6.79 ± 0.31	5.65 ± 0.98	2.81 ± 0.12	1.02 ± 0.39
Observation group (*n* = 35)	7.12 ± 0.39	3.13 ± 0.55	2.97 ± 0.23	0.57 ± 0.02
*t*	0.597	5.559	0.461	5.876
*P*	>0.05	>0.05	>0.05	>0.05

## Data Availability

The dataset used in this paper are available from the corresponding author upon request.
